# A Prediction Model of Health Development Based on Linear Sequential Extreme Learning Machine Algorithm Matrix

**DOI:** 10.1155/2022/7632841

**Published:** 2022-03-07

**Authors:** Suli Cheng, Shuzhi Liu

**Affiliations:** ^1^College of Mathematics and Statistica, Chongqing Technology and Business University, Chongqing 400067, China; ^2^School of Physical Education, Chongqing University, Chongqing 400044, China

## Abstract

The rapid development of social economy not only increases people's living pressure but also reduces people's health. Looking for a healthy development prediction model has become a domestic concern. Based on the analysis of the influencing factors of health development, this paper looks for a model to predict the development of public health, so as to improve the accuracy of health development prediction. In this paper, the linear sequential extreme learning machine algorithm can be used to evaluate the health status of a large number of data, analyze the differences of each evaluation index, and construct the analysis model of health status. Therefore, this paper introduces rough set theory into linear sequential extreme learning machine algorithm. Rough set can analyze the double analysis of evaluation scheme, predict the health development of different individuals, and improve the evaluation accuracy of mass health evaluation. The simulation results show that the improved line sequential extreme learning machine algorithm can accurately analyze the mass health and meet the needs of different individuals' health evaluation.

## 1. Introduction

With the acceleration of the pace of life and the increase of people's work pressure, people pay more and more attention to their health. People pay attention to their own health. Health is divided into subhealth, health, and various diseases. However, due to the individual differences, basic diseases, and their own health quality, the health judgment scheme cannot effectively meet the needs of the public [1]. The survey results show that by 2020, the number of patients with health abnormalities in China will reach 2232/100000, and by 2030, this data will increase by 30%. Among them, 20% of the underground people are unable to take corresponding measures in time due to unreasonable prediction. Therefore, it is an urgent problem to formulate an effective judgment scheme according to personal constitution. Local governments, society, and nongovernmental organizations regularly monitor their health to let the public know their health [2]. At the same time, local governments should also elaborate on the methods of health prediction and publicize them through television, Internet, and other channels. At present, the key of health prediction is how to evaluate relevant indicators and guide different individuals to carry out health test [3]. Some scholars believe that the formulation of health prediction scheme should be combined with personal situation, carry out multiangle regression analysis, and determine the impact of different factors on the test results. Some scholars also believe that the reasonable formulation of health prediction scheme and test plan will enable the public to more accurately understand their health condition; otherwise, it will affect the public's health. At present, there are many methods to analyze mass health, mainly including Bayesian method, genetic algorithm, time series algorithm, and differential evolution algorithm based on vague local search strategy [4]. However, the above algorithm only makes a unified analysis of mass health and cannot realize the differential analysis of different bodies. In order to solve this problem, some scholars put forward the health prediction model based on the combination of rough analysis method and linear sequential extreme learning machine and analyzed the mass health index by using rough set. Rough set method is used to couple the eigenvalues of the data in the health index, and the eigenvalues are extracted by threshold [5], penalty coefficient, weight coefficient, and mean value to obtain more accurate preprocessed data. It can be seen that the linear sequential extreme learning machine algorithm has been applied in the healthy development, but there are few application cases, which need to be further analyzed. Linear sequential extreme learning machine method has the advantage of continuous prediction of healthy development, and rough set has the advantage of massive data processing. The combination of the two can carry out continuous analysis of healthy development prediction. The difference analysis of linear sequential extreme learning machine and its own iterative operation can obtain the optimal set of health data. Among them, the constraint conditions and constraint coefficients can avoid the local extremum problem and improve the efficiency of the calculation results [6]. To sum up, domestic scholars' research on health prediction and analysis mainly focuses on the improvement of indicators, ignoring the coupling between indicators and the rationality of prediction scheme. Therefore, the prediction of healthy development urgently needs a model that can always carry out coupling analysis of various indicators. However, there is less research on continuous prediction of healthy development in China, and there is less research on the application of rough set and linear sequential extreme learning machine. Compared with China, there are many researches on online sequential extreme learning machine abroad, and it is combined with k-clustering and rough set to evaluate the healthy development and achieved good results. So, it is urgent to improve the linear sequential extreme learning machine and apply it to the prediction of healthy development. On this basis, in order to find a more effective model, the improvement of line sequence extreme learning machine and its application to healthy development prediction have become the key to solve the above problems. In addition [7], a single analysis of mass health will not only reduce the accuracy of evaluation results but also affect the future prediction of health. In addition, although the linear sequential extreme learning machine can carry out iterative analysis and predict the mass health, it cannot analyze the individual health. Some scholars believe that the combined analysis of personality and unity can promote the development of health prediction and play a positive role in the improvement of health [8]. Therefore, by optimizing the line sequential extreme learning machine algorithm and combining the rough set processing method, we can accurately evaluate the mass health and obtain the Pareto optimal set. Based on the above theoretical analysis, this paper proposes an improved line sequential extreme learning machine to study mass health [9]. The specific content includes three aspects: the first part introduces the research status of rough set line sequential extreme learning machine and mass health. In the second part, an improved line sequential extreme learning machine algorithm is constructed, and the numerical judgment and constraints of rough set are explained. The third part verifies and analyzes the improved line sequential extreme learning machine algorithm to judge the accuracy and time of mass health calculation [10]. Compared with other studies at home and abroad, this paper optimizes the line sequential extreme learning machine algorithm and combines this method with rough set to obtain the Pareto optimal set under the constraint coefficient [11]. Through the joint analysis of unified health judgment and individual health, we can realize the dual verification of the above two aspects, improve the accuracy of the analysis results, promote the reasonable construction of health evaluation scheme, and finally achieve the purpose of improving mass health.

## 2. The Algorithm Description Based Online Sequential Extreme Learning Machine

The linear sequential extreme learning machine algorithm was first applied to the diagnosis of space engine. It can predict the abnormal situation of aircraft through equal weight processing of data. However, the algorithm cannot realize the analysis of massive data, and the speed of processing massive data is slow. Rough set is a set proposed by Pawlak Z. It can comprehensively process incomplete data through induction, learning, and mining to build a relatively clear and concise data system to support subsequent composition analysis. Based on the above analysis, this paper uses rough set theory to collect mass physical health data [12], supplement incomplete data and indicators, and finally get a clearer data system. The specific data processing flow is shown in Figure 1.

As can be seen from Figure 1, the first step is to obtain physical health data, analyze the data types, and classify them according to the types. The second step is to formulate physical health plan or adjust the plan according to the analysis results of physical health data. The third step is to test the physical health of the masses, compare the effects of different exercise methods, and record the matching results between the exercise scheme and the masses. The fourth step is to record the optimal matching scheme into the database and eliminate the mismatched evaluation scheme. Medical institutions, rehabilitation centers, elderly care centers, sports centers, and fitness centers in four provinces were observed, and preliminary unified data were obtained by means of video recording, heartbeat detection, and vital capacity test. Combined with relevant domestic literature [13], 23 physical health indexes and 12 physical health evaluation indexes are obtained. After experts' determination and 120 sampling questionnaires, there is no significant correlation between the above indexes, which can be used as evaluation indexes and samples. The visit sites are located in the northeast, northwest, southeast, and southwest [14], as well as north and central China. The access data come from online questionnaires, actual data collection, official published materials, and other internal materials. The time span of accessing data is 2–3 years, and the personnel span is more than 4. The validity and reliability of the survey results were >0.7. Finally, specific evaluation indicators are obtained, as shown in Table 1.

## 3. The Prediction Model of Physical Health Development Based on Linear Sequential Extreme Learning Machine Algorithm Matrix Is Established

### 3.1. Improved Line Sequence Extreme Learning Machine Algorithm Matrix

First, add rough sets. In the physical health analysis, the physical health database, physical prediction database, and their correlation database are established by rough set method. Then, rough set uses the above database to analyze the algorithm matrix of linear sequential extreme learning machine and determine the mass constitution. In the process of analysis [15], the weight of different physical health prediction schemes is determined through the correlation, dependence, and correlation between physical health prediction schemes and mass physique. Due to individual differences, basic diseases, knowledge level, and other factors, there are deviations in the impact of the prediction scheme on the prediction results of physical health. Rough set regulates the calculation direction of feature data by setting penalty value, avoids the local extremum problem of line sequential extreme learning machine algorithm matrix, and improves the accuracy of calculation results.

Second, add discrete clustering. The data in rough set present discrete state. Although the weight coefficient is set, it is still unable to realize the continuous analysis of data. How to use finite eigenvalues and feature points to construct continuous rough set sequences is the key of this paper [16]. In this paper, rough set is introduced to classify eigenvalues, and discrete data sequences are constructed by using the correlation and complementarity between adjacent features. At the same time, rough set uses the concept of fuzzy mathematics to eliminate the eigenvalues with high dispersion, calculate the membership relationship between eigenvalues more accurately, and realize the data optimization of linear sequential extreme learning machine algorithm matrix. The improvement process of linear sequential extreme learning machine algorithm matrix is shown in Figure 2.

According to the analysis in Figure 2, rough set analysis is carried out on structured and semistructured data to realize data coupling, fusion, and eigenvalue extraction. Rough set realizes the preprocessing of mass health data. Rough set realizes the orderly arrangement of characteristic data, improves the accuracy of data processing, reduces the data processing time, and increases the amount of preprocessed data.

### 3.2. Analysis of Mass Physical Health Evaluation Scheme Based on Linear Sequential Extreme Learning Machine Algorithm Matrix

In the case of individual differences, the physical health evaluation scheme has a significant impact on the evaluation results, and there are significant differences in the effects of blood oxygen index, blood pressure, and heart rate [17]. Although the linear sequential extreme learning machine algorithm matrix can carry out progressive analysis on mass physical health data, the analysis results are discrete. Rough set can cluster the discrete results, submit the accuracy of the results, and arrange the eigenvalues of the results in order. Rough set can double analyze the physical health scheme and physical data, so as to further improve the accuracy of the results. Therefore, the combination of linear sequential extreme learning machine algorithm matrix and rough set can orderly arrange the characteristic data, improve the accuracy of data analysis results, and realize the double evaluation of mass physical health. The specific evaluation scheme is shown in Figure 3.

It can be seen from Figure 3 that different masses adopt different physical fitness assessment scheme, and different schemes will also have different effects on physical health. Therefore, we should adjust the physical fitness assessment scheme according to the individual differences of masses, so as to achieve the best regulation of physical health.

### 3.3. The Algorithm Construction

#### 3.3.1. Objective Function Construction of Physical Health Evaluation

Assuming that the evaluation objective of physical health is *X*, *y*_*i*_ is the physical fitness assessment scheme, *i* is the exercise program number, and *j* is the correlation between the physical fitness assessment scheme and physical health, *X*_*ij*_ is the evaluation objective of any physical health; the calculation results are shown in

(1) $$\begin{array}{c} \min X=\overset{T}{\underset{\mathrm{i,j}}{\sum }}f\left[x_{ij}\left(1-x_{ij-1}\right)\right]S_{ij}+\varsigma \left(y_{ij}\right), \end{array}$$

where *S*_*ij*_ is the implementation effect of *j* exercise program, *ς*(*y*_*ij*_) is the impact rate of *j* exercise program on physical health, and *T* is the implementation process of physical fitness assessment scheme. *ς*(*y*_*ij*_) is the influence rate of the evaluation scheme; the calculation results are shown in

(2) $$\begin{array}{c} \varsigma \left(y_{ij}\right)=\alpha_{i}+\beta_{i}y_{ij-1}+\chi_{i}y_{j-1}^{2}, \end{array}$$

where *α*_*i*_, *β*_*i*_, and *χ*_*i*_ are the influence coefficients of the evaluation scheme.

#### 3.3.2. Evaluation Function Construction of Aerobic Regimen

It is assumed that the evaluation *H* of aerobic scheme is in three states: scientific and reasonable state *a*_*i*_, vague state *b*_*i,*_ and negative influence state *d*_*i*_; the calculation results are shown in

(3) $$\begin{array}{c} H\left(y_{ij}\right)=\prod \overset{T}{\underset{i=1}{\sum }}A_{ai}+B_{bi}+Cc_{i}. \end{array}$$

Among them, *A*, *B,* and *C* are the evaluation coefficients, and *T* is the time node of different evaluation schemes. The evaluation coefficient is mainly determined by the mass health association, aerobic fitness association, and Chinese Medical Association. At the same time, the evaluation coefficient of each region can be adjusted according to the statistical data of 10 years, and the adjustment proportion is less than 0.3.

#### 3.3.3. Construction of Constraint Function

It is assumed that the upper limit of the evaluation result of physical fitness assessment scheme is *L*max and the lower limit is *L*min. The upper limit of physical health evaluation was *l*max, and the lower limit was *l*min. The calculation results are shown in

(4) $$\begin{array}{c} Z\left(X,H\right)=\overset{\infty }{\underset{\min\approx 0}{\sum }}\frac{\max\left(X,H\right)-{\left(A_{ai}+B_{bi}+C_{ci}\right)}^{\prime }}{{\left(A_{ai}+B_{bi}+C_{ci}\right)}^{\prime }-\min\left(X,H\right)}\prod_{\min}f\left[x_{ij}\left(1-x_{ij-1}\right)\right]S_{ij}^{\prime }, \end{array}$$

where max(*X*, *H*) is the maximum value set of evaluation results, min(*X*, *H*) is the minimum value set of evaluation results, and (*A*_*ai*_+*B*_*bi*_+*C*_*ci*_)′ is any maximum value. *S*_*ij*_′ is optimal physical fitness assessment scheme. The specific construction process is shown in Figure 4.

It can be seen from Figure 4 that the calculation process of physical fitness assessment scheme and physical health prediction exceeds the expected maximum and minimum values, indicating that the setting of constraints can limit the differential evolution process of vague local search strategy. At the same time, the physical fitness assessment scheme and the improvement of physical health did not change significantly, showing regular ups and downs. At the same time, the following picture in Figure 4 shows a large depression, indicating that the data here are an inflection point. However, the data in the depression still changes smoothly, which further shows that the data processing effect is better.

### 3.4. The Construction of Linear Sequential Extreme Learning Machine Algorithm Matrix

The linear sequential extreme learning machine algorithm matrix based on vague local search strategy is mainly in three aspects. The calculation results are shown in

(5) $$\begin{array}{c} \left|E\right|=Z\left(\cdot \right)\times \overset{⌢}{\left\{\begin{array}{c} \overset{n}{\underset{\mathrm{i,j}=0}{\sum }}\underline{x_{ij}},\underline{y_{ij}}\\ \overset{n}{\underset{i=0}{\sum }}S_{j}^{H\left(\text{(}2\pi /2\right)\left(x_{ij},y_{ij}\right)} \end{array}\right.}, \end{array}$$

where $\underline{x_{ij}}$ and $\underline{y_{ij}}$ are the approximate set of *x*_*ij*_ and *y*_*ij*_, and |*E*| is the coupling set. *i* ≠ *j*, *i*, *j* ∈ {1, ⋯, *n*}, ∪_*i*,*j*=1_^*n*^*X*_*ij*_, *H*_*ij*_=*U*. *U* is the correlation between *X*_*ij*_ and *H*_*ij*_ . The second aspect is to cluster discrete eigenvalues by using rough set method to reduce the discreteness of eigenvalues. The specific formula is as follows.

Assuming the sample set *X*={*x*_11_, *x*_12_ ⋯ *x*_*ij*_}, *H*={*h*_11_, *h*_12_ ⋯ *h*_*ij*_}, the clustering center *V* of each dimension is shown in

(6) $$\begin{array}{c} V=\left\{v_{11},v_{12}\cdots v_{ij}\right\}. \end{array}$$

The membership matrix *u* of each cluster center *V* is shown in the formula. The calculation results are shown in

(7) $$\begin{array}{c} u=\left[\begin{array}{cccc} u_{11} & \cdots & \cdots & u_{1j}\\ \vdots & \ddots & \; & \;\\ \; & \; & \; & \vdots \\ u_{i1} & \; & \; & u_{ij} \end{array}\right], \end{array}$$

where *u*_*ij*_ is the subordinate relationship between the sample *u*_*i*_ and *u*_*j*_. The formula of rough set function is shown in

(8) $$\begin{array}{c} \min F\left(u_{ij},v_{i}\right)=\underset{i=1}{\sum }\underset{j=1}{\sum }u_{ij}^{\tau }\left(x_{ij}-v_{i}\right), \end{array}$$

where *τ* is the clustering index between *X*_*ij*_ and *H*_*ij*_. The calculation of *v*_*i*_ cluster center is shown in

(9) $$\begin{array}{c} v_{i}=\frac{x_{ij}}{\sum_{i=1}u_{ij}^{\tau }\left(x_{ij}-v_{i}\right)}\sum u_{ij}^{\tau }\left(x_{ij}-v_{i}\right). \end{array}$$

The calculation of membership relationship is shown in

(10) $$\begin{array}{c} u_{ij}=\frac{{\left(1/\Delta x_{ij}\right)}^{1/\left(\tau -1\right)}}{\sum_{i=1}{\left[1/\left(\Delta x_{ij}-v_{i}\right)\right]}^{1/\left(\tau -1\right)}}. \end{array}$$

The third aspect is to determine the weight coefficient. In order to more accurately analyze the physical fitness assessment scheme and realize the comprehensive evaluation of the impact of physical health [18], the weight of each index should be assigned. At the same time, the weight assignment can avoid the local extreme value problem and improve the accuracy of the evaluation results. Firstly, each objective function is regarded as a conditional attribute [19], its weight is obtained, and the optimal template function *X* value is calculated. Secondly, the evaluation template attribute set is obtained [20]. The optimal scheme obtained under different physical fitness assessment scheme is *h*; then, any physical fitness assessment scheme in *X* is *u*_*ij*_.

Therefore, the dependence between physical fitness assessment scheme and physical health evaluation is shown in the formula. Firstly, each objective function is regarded as a conditional attribute, *w*_*i*_=1/*n*_*i*_ weight is obtained, and the optimal template function *X* value is calculated. Secondly, the evaluation template attribute set *D*={*X*} is obtained. The optimal scheme obtained under different physical fitness assessment scheme is *H*; then, any physical fitness assessment scheme in *X* is *u*_*i*_,.

Therefore, the dependence between physical fitness assessment scheme and physical health evaluation is shown in

(11) $$\begin{array}{c} r_{i}\left(H\right)=\frac{\sum \rho \left[r_{i}{\left[F\right]}_{D}\right]}{\rho \left(u_{i}\right)}. \end{array}$$

The degree of dependence between evaluation objectives is shown in

(12) $$\begin{array}{c} \Delta r_{i}\left(H\right)=\frac{\sum \rho \left[\Delta r_{i}{\left[F\right]}_{D}\right]}{\rho \left(\Delta u_{i}\right)}. \end{array}$$

The importance of the *i*th physical health assessment is shown in

(13) $$\begin{array}{c} \sigma \left(X,H\right)=r_{i}\left(H\right)-\Delta r_{i}\left(H\right). \end{array}$$

The weight between the *i*th physical health assessment and physical health is shown in

(14) $$\begin{array}{c} w_{i}=\sigma \left(X_{i},H_{i}\right)/\sum \sigma \left(X,H\right). \end{array}$$

In order to give weight more accurately, increase the residual value of weight change. The calculation results are shown in

(15) $$\begin{array}{c} w_{i}=\sigma \left(X_{i},H_{i}\right)/\sum \sigma \left(X,H\right)+\xi , \end{array}$$

where *ξ* is the residual value of weight, which is mainly determined by the development of physical health in different regions.

### 3.5. The Output of Physical Health Evaluation Results under Linear Sequential Extreme Learning Machine Algorithm Matrix

Firstly, the physical fitness assessment scheme output of different individuals: physical health is multidimensional, complex, and irregular, so it is affected by individual physical quality, basic diseases, training methods, training time, and other factors.

Assuming that different influence factors are *k*_*i*_, the output of physical fitness assessment scheme under different factors is shown in

(16) $$\begin{array}{c} H{\left(y_{ij}\right)}_{k}=v_{i}\cdot \prod_{k}\lambda \cdot \overset{T}{\underset{i=1}{\sum }}A_{ai}+B_{bi}+Cc_{i}, \end{array}$$

*v*_*i*_ is the data after rough set, *k* is the influencing factor, *H*(*y*_*ij*_)_*k*_ is the output optimal physical fitness assessment scheme, and *λ* is the differential evolution coefficient. Therefore, the application of rough set method improves the adaptability of physical fitness assessment scheme, meets the exercise needs of different individuals, and realizes the effective aggregation of discrete eigenvalues.

### 3.6. Physical Health Evaluation Output of Different Physical Fitness Assessment Schemes

Different physical fitness assessment schemes have different effects on physical health, so it is necessary to accurately evaluate physical health. Generally speaking, the improvement of physical health is judged in the form of ten-point system. Under the action of rough set, the output results of physical health evaluation are calculated. The calculation results are shown in

(17) $$\begin{array}{c} X_{H_{i}}=\overset{⟶}{\frac{w_{i}\cdot \varsigma \left(y_{ij}\right)\sum_{i,j}^{T}f\left[x_{ij}\left(1-x_{ij-1}\right)\right]S_{ij}+\varsigma \left(y_{ij}\right)}{v_{i}\cdot \prod_{k}\lambda \cdot \sum_{i=1}^{T}A_{ai}+B_{bi}+Cc_{i}}}, \end{array}$$

where *H*_*i*_ is different physical fitness assessment scheme and *λ* is the coefficient of differential evolution.

Secondly, the calculation steps of physical health evaluation results. Through the above analysis, the overall overview of physical health analysis can be obtained. The specific steps are as follows.

First, construct a rough set of the impact of such exercise on physical health, and form *X*={*x*_11_, *x*_12_ ⋯ *x*_*ij*_} and *H*={*h*_11_, *h*_12_ ⋯ *h*_*ij*_} sets.

Secondly, the data set is constrained, the clustering center V of the data is calculated, the weights of physical fitness assessment scheme and physical health are obtained, and the corresponding iterative operation is carried out. If the calculation results *X* and H are greater than max{*X*, *H*}, the results shall be included in the calculation results; otherwise, they shall be eliminated. If the calculation result is less than min{*X*, *H*}, the result shall be included in the calculation result; otherwise, it shall be eliminated.

Third, when all 35 indicators are traversed, output *H*(*y*_*ij*_)_*k*_, *X*_*H*_*i*__; otherwise, repeat Step 2.

## 4. The Cases of Physical Health Assessment and Prediction

### 4.1. The Research Data through the 35 Indicators Obtained from the Survey: A Case Study Is Carried Out

The data in the case mainly comes from 6 randomly selected cities, and the verification method is mainly to compare before and after (note: the validity and reliability of the data are >0.7) [21]. At the same time, the linear sequential extreme learning machine algorithm matrix is compared with the original algorithm (note: linear sequential extreme learning machine algorithm is not combined with rough set). The verification period is January, March, June, and December, and the exercise intensity is 60 H/week. The subjects were 25–65 years old, with an average age of 32.2 ± 2.32 years [22]; BMI 23–40, average BMI 28.2 ± 1.12. Inclusion criteria: (1) Meet the 1994 edition of American diagnostic criteria for physical health. (2) The subjects had no previous physical health and circulatory diseases. (3) Get the consent of the ethics committee of the hospital and sign the informed consent form. (4) The tester can express himself. (5) The tester has some fitness experience. The results are shown in Table 2.

The data in Table 2 are the evaluation contents in different test time periods, mainly including training intensity and training score, and the data are from the experimental results and network literature. In order to ensure the accuracy of the test, the tester should be analyzed before the test. According to different methods, they were divided into improvement group and original group. The improved group adopts the differential evolution algorithm of improved vague local search strategy, and the original group adopts the differential evolution algorithm of vague local search strategy. The results are shown in Table 3.

It can be seen from Table 3 that there is no significant difference between the two groups in physical health, pulmonary respiratory capacity, blood pressure, quality of life, blood oxygen content, and pulse, so it can be compared and analyzed.

### 4.2. Evaluation of Physical Fitness Assessment Scheme by Linear Sequential Extreme Learning Machine Algorithm Matrix

The accuracy of physical fitness evaluation scheme evaluation is the key of evaluation. The linear sequential extreme learning machine algorithm improves the fuzzy local search strategy. The specific evaluation results are shown in Figure 5.

It can be seen from Figure 5 that the average accuracy of physical fitness assessment scheme is more than 90%, and the effective scheme is more than 60%. At the same time, the effective program of physical health was the highest at 96% and then decreased. The results of this study are consistent with relevant domestic studies. The reason is that after the human physical health reaches the maximum limit, the body's self-protection mechanism starts, resulting in a decline in the improvement of physical health. The linear sequential extreme learning machine algorithm matrix is compared with the original algorithm, and the results are shown in Figure 6.

It can be seen from Figure 6 that the linear sequential extreme learning machine algorithm matrix has high evaluation accuracy of physical health, greater than 99%, while the accuracy of the original algorithm is greater than 90%; the results of this study are consistent with relevant domestic studies. This shows that the linear sequential extreme learning machine algorithm matrix is better in physical fitness assessment scheme. It can be seen from the figure that the evaluation results of the two methods change smoothly. However, the model proposed in this paper changes straightly, while the original line sequence extreme learning machine algorithm changes at the positions of the 4th, 6th, 11th, 13th, 16th, 22nd, 24th, 26th, 28th, 32^nd^, and 33rd times. Therefore, the model proposed in this paper is better.

### 4.3. The Evaluation of Physical Health by Linear Sequential Extreme Learning Machine Algorithm Matrix

Physical health evaluation is the computational goal of differential evolution algorithm to improve vague local search strategy, and it is also an effective embodiment of physical health calculation. The evaluation results of physical health are shown in Figure 7.

It can be seen from Figure 7 that the changes of 35 physical health evaluation indexes are relatively stable, indicating that the contribution rate of physical health indexes under different algorithms is relatively stable, which verifies the effectiveness of physical health indexes; the results of this study are consistent with relevant domestic studies [23]. At the same time, the evaluation result of physical health under the linear sequential extreme learning machine algorithm matrix is better, and its change range gradually reduces to 100%. In contrast, the differential evolution algorithm based on vague local search strategy has not changed, and the result is about 7%. The reason is that the rough set method improves the index aggregation of physical health, provides effective physical fitness assessment schemes for different individuals, and realizes the significant improvement of physical health. Although the differential evolution algorithm of vague local search strategy also provides evaluation scheme for physical health, in the case of randomness, physical fitness assessment scheme presents beneficial and unhelpful changes, resulting in the final improvement of 7%.

### 4.4. The Coupling between Physical Fitness Assessment Scheme and Physical Health

The coupling between physical fitness assessment scheme and physical health is not only the advantage of differential evolution algorithm to improve vague local search strategy, but also the result of two-way evaluation. For better analysis, linker analysis method is selected (uncoupled, general coupling, general, coupling, and comparative coupling, with values of 1–7 respectively). The calculation results are shown in Figure 8.

As can be seen from Figure 8, the coupling between physical fitness assessment scheme and physical health shows an upward trend and approaches the value of 5, indicating that the coupling between the two is better. The results of this study are consistent with relevant domestic studies [24]. Relatively speaking, the linear sequential extreme learning machine algorithm matrix has better coupling, which is significantly better than the differential evolution algorithm with vague local search strategy. The above results also show that rough set can greatly improve the coupling of linear sequential extreme learning machine algorithm matrix and realize the two-way evaluation of physical fitness assessment scheme and physical health. In order to further verify the coupling results, 35 specific indicators are analyzed, and the results are shown in Figure 9.

It can be seen from Figure 9 that the coupling of 35 indicators is better. The results of this study are consistent with relevant domestic studies. Among them, the linear sequential extreme learning machine algorithm matrix has better coupling [Note: 24 red indicators], and the coupling under the two algorithms meets the maximum and minimum constraints of penalty value.

## 5. Conclusion

At present, the research on the impact of physical health on subdivision function has the problem of single evaluation [25], which cannot realize the dual evaluation of physical fitness assessment scheme and the improvement of physical health, so that physical fitness assessment scheme cannot effectively improve physical health. Therefore, how to effectively use physical fitness assessment scheme to improve people's physical health and realize national fitness is an urgent problem to be solved. Based on this background, this paper improves the differential evolution algorithm of vague local search strategy and integrates the rough method set to realize the dual evaluation of physical fitness assessment scheme and physical health. In this paper, firstly, rough set is used to calculate the eigenvalues of physical fitness assessment scheme and physical health evaluation, then rough set is used to eliminate redundant data, and finally the dual evaluation of physical fitness assessment scheme is done. In order to submit the accuracy of evaluation, the constraint conditions and penalty values of rough set are set. MATLAB simulation results show that the linear sequential extreme value learning machine algorithm matrix combined with rough set has a good effect on physical health evaluation and prediction. The result accuracy is greater than 95% and the fitting degree is 98%, which is better than the result of linear sequential extreme value learning machine algorithm matrix. Therefore, using linear sequential extreme value learning machine algorithm matrix combined with rough set can realize physical health evaluation and prediction, improving the accuracy of the results. However, the interaction between physical health assessment and prediction is not analyzed in the process of rough set analysis in this paper. This aspect will be emphatically analyzed in future research.

## Figures and Tables

**Figure 1:** The data processing process of physical health development prediction.

**Figure 2:** The physical health assessment scheme and prediction.

**Figure 3:** The implementation process of linear sequential extreme learning machine algorithm matrix.

**Figure 4:** The constraint analysis of physical fitness assessment scheme and physical health prediction.

**Figure 5:** The evaluation results of physical health.

**Figure 6:** The evaluation results of physical health under different algorithms.

**Figure 7:** The physical health evaluation results.

**Figure 8:** The coupling of physical health regimen and physical health.

**Figure 9:** The coupling of physical health regimen and different indexes of physical health.

**Table 1:** The mass physique and health evaluation index.

The index category		The quantity	The correlation with other indicators
Amount of exercise	Type of motion	4	0.232
	Exercise time	3	0.767
	Exercise intensity	2	0.562

Body function	Blood oxygen content	9	0.222
	Respiratory rate	4	0.721
	Cardiac blood supply	6	0.492
	Lung volume	3	0.662
	Inflammatory factor index	2	0.892

*Note.* There is no significant correlation between the indicators, and the reliability and validity are >0.7. The data come from online literature and actual survey.

**Table 2:** The evaluation contents of test.

Duration	1∼2 h	2–2.3 h	1–3.2 h	1∼2 h	1–1.5 h	1–1.5 h	1∼2 h	1∼3 h
Exercise time	300 KJ	4333 KJ	1222 KJ	4333 KJ	2392 KJ	1223 KJ	4303 KJ	2322 KJ
Exercise intensity	1–5	7–11	9–22	11–19	33–89	102–111	47–82	46–90
Physical health score	10 score	10 score	10 score	10 score	10 score	10 score	10 score	10 score
Physical health degree	3	1	3	2	1	1	2	1

**Table 3:** The comparison of pretest indexes of masses [n, $\bar{x}$ ±*s*].

The group	Physical health score (score)	Physique index (piece)	Blood pressure (cm H2O)	Physical fitness standard rate (%)	Quality of life score (m3/ml)	Pulse (mmHg)
Improvement group (*n* = 20)	6.33 ± 5.21	28.61 ± 6.42	78.34 ± 5.27	88.71 ± 6.22 *∗*	186.49 ± 11.24 *∗*	70.13 ± 9.82 *∗*
Original group (*n* = 20)	6.84 ± 5.32	28.97 ± 6.53	78.52 ± 5.42	87.42 ± 6.97 *∗*	179.14 ± 7.27 *∗*	73.62 ± 8.14 *∗*
*T*	0.907	0.176	0.107	0.192	0.137	0.789
*P*	0.370	0.861	0.916	0.893	0.726	0.822

## Data Availability

The data used to support the findings of this study are available from the corresponding author upon request.
